The article "Tumor-suppressive miR-26a and miR-26b inhibit cell aggressiveness by regulating FUT4 in colorectal cancer" was published in 2017. Journal: Cell Death Dis.

# Tumor-suppressive miR-26a and miR-26b inhibit cell aggressiveness by regulating FUT4 in colorectal cancer

**DOI:** 10.1038/cddis.2017.281

**Published:** 2017-06-22

**Authors:** Yang Li, Zheng Sun, Bing Liu, Yujia Shan, Lifen Zhao, Li Jia

**Affiliations:** 1 College of Laboratory Medicine, Dalian Medical University, Liaoning Province, Dalian 116044, China

## Abstract

Metastasis is a multistep molecular network process, which is the major cause of death in patients with colorectal cancer (CRC). MicroRNAs (miRNAs) play pivotal roles in tumorigenesis as either tumor suppressors or oncogenes. Increased expression of fucosyltransferase4 (FUT4) has been reported to be associated with the invasive and metastatic properties of CRC. Here to identify potential key miRNAs and their target genes for colorectal cancer (CRC), we compared miRNA expression profiles between metastatic CRC cell SW620 and primary CRC cell SW480. Microarray analysis revealed that there were 85 differentially expressed miRNAs in SW620 cells with highly metastatic potential compared to SW480 cells with lowly metastatic potential. The expression of miR-26a and miR-26b were lower in SW620 cells than in SW480 cells, as well as downregulated in tumor tissues than in adjacent normal tissues of CRC patients. By applying bioinformatic approaches for the prediction of miRNA targeting 3′-UTR of FUT4, we identified FUT4 as one of the miR-26a/26b-targeted genes, while the expression of the target gene exhibited patterns opposite to that of miR-26a/26b in CRC cell lines, tumor tissues and corresponding adjacent tissues. Forced miR-26a/26b expression affected migratory behavior of CRC cells and FUT4 expression, while altered expression of FUT4 in CRC cell lines modulated progression upon transfection with miR-26a/26b mimic or inhibiter. FUT4 also regulated directly aggressiveness of SW620 and SW480 cells. Moreover, statistical analyses revealed that low miR-26a/26b levels and high expression of FUT4 were positively correlated with poor overall survival. The identified CRC-restricted miR-26a and miR-26b might be implicated in cancer progression via their target gene FUT4, suggesting their potential usage in CRC treatment.

As one of the most common malignant cancers worldwide, colorectal cancer (CRC) has become the fifth leading cause of cancer death for men and women in China.^1^ Altough the CRC stage at diagnosis is the most predictive factor of clinical outcome, the remaining 20–30% of newly diagnosed CRC patients is unresectable distant metastasis.^2^ Survival rates are highly dependent on the occurrence of distant metastases.^3^ Therefore, a better understanding of the molecular mechanisms involved in CRC metastasis will provide diagnostic and prognostic markers and potential targets for the therapeutic intervention of CRC metastasis.

MicroRNAs (miRNAs) are 18–22 nucleotide non-coding RNAs that post-transcriptionally regulate gene expression and control various cellular mechanisms including tumorigenesis and the development of various types of cancers.^4, 5, 6^ Bioinformatics and cloning studies have indicated that miRNAs may post-transcriptionally regulate almost 60% of all human genes and control hundreds of cognate gene targets through their oncogenic or tumor-suppressive activity.^7^ Recent studies have shown the altered expression of miRNAs during the development of colorectal cancer, highlighting their potential for diagnostic and prognostic applications, and classification of human malignancies.^8, 9, 10^ Given the extensive role of miRNAs in gene regulation and cellular processes, the evaluation of miRNAs as regulators of tumor aggressiveness and prognosis is of interest.^11, 12^ Since miRNAs are very resilient against degradation, they are considered a powerful diagnostic tool.

Glycosylation is a common and highly diverse form of protein modification,^13, 14^ and plays a pivotal role in many biological processes. The glycosylation form and density of glycans on a protein can be altered significantly in association with changes in cellular pathways and processes resulted from diseases, such as malignancy. Several CRC tissue-associated changes in glycans have been reported and recently reviewed.^15^ Holst *et al.*^16^ showed pronounced differences between the *N*-glycosylation patterns of CRC cell lines, and CRC cell line profiles differed from tissue-derived *N*-glycan profiles. Osuga *et al.*^17^ found that increased fucosylation was correlated with metastatic potential in CRC. Investigation of CRC-associated fucosylation changes can be vital for better understanding of the function of fucosyltransferases (FUTs) in the progression of CRC.

The fucosyltransferase FUT4 is capable of catalyzing the fucosylation of glycoproteins. FUT4 was highly expressed in gastric cancer tissues and serum, respectively as compared to chronic gastritis and gastric ulcer.^18^ FUT4 was a novel regulator of epithelial–mesenchymal transition (EMT), which was a crucial step in tumor progression in breast cancer cells.^19^ FUT4 was also overexpressed in most of metastatic colorectal cancer patients and associated with poorer outcomes.^20^ In our previous studies, the altered level of FUT4 was responsible for changed drug-resistant phenotypes of human hepatocellular carcinoma (HCC) cell lines BEL7402 and BEL/FU cells both *in vitro* and *in vivo*.^21^ Although FUT4 is well-known to play an important role in cancer progression, the underlying mechanisms of fucosylation mediated by miRNA remain unknown in CRC.

In the present study, to further strengthen the clinical application of miRNAs and FUT4 for the diagnosis of CRC progression, we first performed a discovery step based upon miRNAs and FUT4 with published evidence as potential diagnostic biomarkers of CRC.

## Results

### MiRNA expression profile in SW620 and SW480 cells

To test whether these epigenetic differences are associated with changes in the level of miRNA expression and to investigate the role of miRNA in the development of metastasis, we analyzed the miRNA expression profiles of SW620 cells with highly metastatic potential and SW480 cells with lowly metastatic potential. The microarray analysis revealed significant changes in miRNA expression profile in SW620 cells compared to SW480 cells.

The results showed 85 miRNA genes (33 up-regulated and 52 down-regulated) that were differentially expressed in SW620 cells compared with SW480 cells (Figure 1a). Fold change greater or equal to 2 have been considered as significant change. Among these significantly differentially expressed miRNAs, 2 tumor suppressor miRNAs (miR-26a and miR-26b) were further validated individually using qRT–PCR. The results of qRT–PCR confirmed the miRNA array results whereby the expression level of the selected miRNA was lower in the SW620 cells than the SW480 cells (Figure 1b). Similar significant findings were identified in CRC samples (Figure 1c). MiR-26a/26b expression was significantly decreased in 38 pairs of CRC tissues compared to adjacent tissues by qRT-PCR. Because the expression of miR-26a and miR-26b was markedly decreased in CRC tissue samples and SW620 cells with highly metastatic potential, they were considered important miRNAs for colorectal tumor progression. Therefore, we focused our efforts on the identification of candidate oncogene regulated by miR-26a/26b.

### Identification of FUT as a target of miR-26a and miR-26b in CRC

It is well known that a single miRNA can affect multiple targets via distinct mechanisms. To study the mechanisms responsible for CRC progression, we performed bioinformatics analyses to search for miR-26a and miR-26b target mRNAs. Bioinformatics tools revealed potential binding sites for miR-26a and miR-26b in FUT4 gene. To further verify that miR-26a and miR-26b directly target the 3′UTR of FUT4, direct interaction between miR-26a/26b and the 3'UTR from FUT4 was subsequently validated using a luciferase-based assay. The luciferase activity of the reporter construct containing the wild-type FUT4 3′-UTR was repressed by miR-26a/26b mimic, whereas these miRNAs had no effect on the luciferase activity of reporter constructs containing mutant FUT4 3′-UTR (Figure 2a). These results implicate that FUT4 is a direct target gene of miR-26a and miR-26b.

We next examined whether FUT4 expression is regulated by endogenous miR-26a and miR-26b in CRC cell lines. As shown in Figures 2b and c, SW620 cells were transfected with miR-26a or miR-26b mimic, SW480 cells were transfected with inhibitor and FUT4 expression levels were measured. Exogenous overexpression of miR-26a and miR-26b decreased the mRNA and protein levels of endogenous FUT4 in SW620 cells (Figure 2b). Conversely, inhibition of miR-26a and miR-26b significantly increased FUT4 levels in SW480 cells (Figure 2c). Immunofluorescence analysis showed that FUT4 antigen expression was significantly decreased in SW620 cells treated with miR-26a/26b mimics, and increased in SW480 cells treated with miR-26a/26b inhibitor (Figures 2d and e). Furthermore, analysis of miR-26a/26b and FUT4 expression in CRC patients showed a significant inverse correlation (*P<0.01; Figure 2f), suggesting that miR-26a and miR-26b was a relevant contributing alteration to regulate FUT4 in CRC patients. The results were consistent with CRC cell lines. Compared to expression in SW480 cells, FUT4 levels were upregulated (Figure 2g) and miR-26a/26b was downregulated in SW620 cells. IHC staining also showed FUT4 expression was significantly up-regulated in SW620 cells as compared with SW480 cells, and in CRC tissues as compared with adjacent tissues (Figure 2h). Together, the results reveal a network of cancer-associated FUT4 that is controlled by miR-26a/26b in CRC.

### MiR-26a/26b impairs aggressiveness of SW620 and SW480 cells in a FUT4-dependent manner

To investigate the potential role of miRNA-mediated down-regulation of FUT4 affecting proliferation and invasion in CRC cells, SW620 and SW480 cells were transfected with either miR-26a/26b mimic or inhibitor. Interestingly, CCK-8 assays revealed that SW620 cells in the miRNA mimic groups had lower proliferative ability and colony formation efficiency than controls (Figures 3a and c). The miR-26a/26b- downexpressing SW480 cells showed higher proliferation and colony formation efficiency compared with the negative control (Figures 3a and d). In support of this idea, the proliferation biomarker Ki67 was assessed. The cells infected with miR-26a/26b mimic showed a decrease level of Ki67, whereas knockdown of miR-26a/26b had the opposite effect on Ki67 expression (Figure 3b). The wound-healing assay showed that the gap between the scorings was larger in mimic-treated group than in control group in 48 h (Figure 3e). By contrast, we observed shorter distance in wound healing of miRNA inhibitor groups compared with control groups (Figure 3f). In cell invasion assays, exogenously upregulation of miR-26a/26b expression significantly inhibited the number of invasive cells significantly (Figure 3g). In addition, increased effects on cell invasion were found by anti-miR-26a/26b in SW480 cells (Figure 3h). These results indicate that miR-26a and miR-26b, which target FUT4, play a role in CRC cell progression.

To next assess whether FUT4 reverses the effect of miR-26a and miR-26b-mediated CRC cell progression, we modulated the expression of FUT4 in SW620 and SW480 cells ectopically expressing miR-26a and miR-26b. Western blot analysis showed overexpression of ST8SIA4 in SW620 cells led to a marked increase in the protein expression upon transfection with miR-26a/26b mimic compared to control (Figures 4a and b). Of importance, we also observed that ectopic expression of FUT4 significantly restored cell colony formation and invasion in SW620 cells transfected with miR-26a/26b mimic compared to control (Figures 4c and d). On the other hand, the results showed that depletion of FUT4 in SW480 cells by an RNAi-mediated silencing approach led to a marked decrease in FUT4 levels upon transfection with the miR-26a/26b inhibitor (Figures 4e and f). Interestingly, we observed that knockdown of FUT4 expression was able to reverse miR-26a/26b inhibitor-mediated colony formation and invasion in SW480 cells (Figures 4g and h). Altogether, these results would indicate that FUT4 regulation is a key event which mediates miR-26a and miR-26b-induced antitumor effects in CRC.

### FUT4 regulates aggressiveness of SW620 and SW480 cells

Because miR-26a and miR-26b directly regulated the expression of FUT4, we examined whether FUT4 would also exert a direct regulation on the response to CRC aggressiveness. SW620 cell line was subjected to FUT4 knockdown and showed a lower level of FUT4 compared with those in the controls (Figure 5a). The down-regulation of FUT4 inhibited SW620 cell proliferation (Figure 5b), invasion and tube formation (Figures 5b–d). The effect of FUT4 on the tumorigenic potential of SW620 cells was investigated *in vivo*. FUT4 shRNA exerted a negative effect on the tumorigenic potential of SW620 cells (Figure 5e). IHC staining also showed the regulatory role of FUT4 shRNA on the expression of FUT4 and Ki67 in the tumor tissues (Figure 5f).

SW480 cell line stably expressing wild type FUT4 showed the enhanced expression of FUT4 to control (Figure 5g). The overexpression of FUT4 in SW480 cells showed that FUT4 indeed regulated SW480 cell proliferation, invasion and tube formation (Figures 5h–j). The *in vivo* injection of wild type FUT4 increased the tumorigenic potential of SW480 cells (Figure 5k). IHC staining showed higher expression of FUT4 and Ki67 in SW480/FUT4 cells compared with those in the controls (Figure 5l). Taken together, these results suggest that miR-26a and miR-26b regulate the aggressiveness of CRC cells in a manner associated with the expression regulation of FUT4.

### Clinical significance of miR-26a/26b downregulation and FUT4 upregulation in CRC

We next investigated the potential clinical significance of miR-26a/26b and FUT4 in CRC. Clinical follow-up data were available for all the 58 patients included in the study. Of relevance, we found that those patients with low miR-26a and miR-26b expression showed a substantially shorter overall survival (miR-26a: HR: 7.697, 95% CI: 3.72-15.92, *P<*0.001; miR-26b: HR: 6.31, 95% CI: 2.90-13.72, *P<*0.001) (Figures 6a and b). As expected, we confirmed that those patients with FUT4 overexpressed showed a substantially shorter overall survival (HR: 6.13, 95% CI: 32.99-12.58, *P<*0.001; Figure 6c).

We next stratified our cohort by miRNA status, observing that miR-26a/26b showed an increased risk of death in those patients with downregulated miR-26a/26b than in those cases with upregulated miR-26a/26b (*P<*0.05, Tables 1 and 2). Subsequently, we found that increased stage (*P*=0.037) and high levels of FUT4 were correlated with an increased risk of death (Table 3). In contrast, there was no significant association between miR-26a/26b, FUT4 expression and prognosis in the age and gender (Tables 1, 2 and 3). Overall, these data suggest that the levels of miR-26a and miR-26b may be associated with overall survival of FUT4-expressed CRC patients.

## Discussion

In the present study, we identified that expression of miRNAs was significantly different between CRC cell line SW620 and SW480 with different metastatic potential. Among them, low-level expression of miR-26a and miR-26b was detected in tumor tissues and highly metastatic CRC cells. Furthermore, miR-26a/26b regulated CRC progression partly through targeting FUT4, while altered expression of FUT reversed the function. Finally, The differential levels of miR-26a/26b and FUT4 were associated with clinical significance of CRC. This is the first study that miR-26a/26b inhibit cell aggressiveness by regulating FUT4 in CRC.

Cumulative evidence revealed a functional involvement of dysregulated miRNAs in cellular alteration, oncogenesis,and survival of CRC cases.^22^ Our current work on CRC revealed multiple miRNA–mRNA regulatory networks, and had proposed loss and gain of some miRNAs as a key mechanism leading to CRC development and progression. Microarray data showed 85 miRNA genes (33 upregulated and 52 downregulated) that were differentially expressed in human CRC cell lines SW620 and SW480, which had high and low potentials of metastasis. Several of the deregulated miRNAs identified in the current study have been reported previously, suggesting a common underlying molecular mechanisms leading to CRC progression. Similarly, we identified miR-26a and miR-26b to be downregulated in SW620 cell line and CRC tissues in our data, which were also reported to be downregulated in CRC patients and CRC cell lines.^23, 24^ These results additionally demonstrate that miR-26a and miR-26b represent potential therapeutic targets to treat CRC metastasis.

MiRNAs have recently emerged as key regulators of cancer development and progression by targeting multiple cancer-related genes. A few miRNAs that target fucosylation enzymes have been identified so far. Wang *et al* reported that miR-198 targeted the 3′UTR of FUT8 directly to downregulate FUT8 expression at both mRNA and protein levels in CRC.^24^ Also FUT8 was identified as a direct target for miR-122 and miR-34a in hepatocarcinoma cell line,^25^ and FUT2 was found a target for miR-15b.^26^ We recent research showed that miR-26a, miR-34a and miR-146a directly targeted FUT8 expression in human hepatocellular carcinoma,^27^ as well as FUT6 was directly targeted by miR-106b in human breast cancer.^28^ FUT4 was found as a novel direct target of miR-224-3p, and the association of FUT4 expression with miR-224-3p was validated in breast cancer mouse models and cell lines.^29^ Furthermore, miR-493-5p directly targeted and inhibited FUT4 expression in breast cancer.^30^ In the current study, *in silico* prediction has identified miR-26a and miR-26a targeting FUT4 in CRC cells, and forced expression of miR-26a and miR-26a phenocopied the effects of FUT4 depletion in CRC cell lines, supporting a role of the two miRNAs in regulating FUT4 expression in CRC. Furthermore, we observed significant inverse relationship between miR-26a and miR-26a and FUT4 expression in 38 pairs of CRC tissues, corroborating the biological relevance of this regulatory network in CRC.

Our current study corroborated previous studies that reported biological effects of miR-26a and miR-26b in CRC progression. However, these studies have identified a different set of target genes. Konishi *et al.*^23^ reported that miR-26a suppressed the progression CRC through inhibition of the binding of Heterogeneous ribonucleoprotein A1 (hnRNP A1)—cyclin dependent kinase 6 (CDK6). Chen *et al.*^31^ reported that miR-26a-regulated glucose metabolism, which has been an emerging hallmark of cancer cells, by direct targeting PDHX in CRC cells. Over expression of miR-26b strongly inhibited CRC cell survival and invasion by direct targeting Nicotinamide phosphoribosyl transferase (Nampt).^32^ Here our results additionally demonstrated the function of miR-26a/26b in regulating progression of CRC cell lines might be partially mediated through targeting FUT4. Overexpression of miR-26a/26b resulted in the inhibitory effects in SW620 cell growth and invasion. In contrast, inhibition of miR-26a/26b might stimulate the proliferative and invasive ability of SW480 cells. Moreover, we found that overexpression of FUT4 significantly restored cell proliferation and invasion in SW620 cells transfected with miR-26a/26b mimic. Knockdown of FUT4 reversed the stimulative effects of miR-26a/26b inhibition in SW480 cell growth and invasion. FUT4 has been regarded as a cancer-related fucosyltransferase and accumulating evidence demonstrated its crucial roles in the development of cancer. For example, FUT4 was overexpressed in most of metastatic colorectal cancer (mCRC) patients (43%), and participated in cetuximab or bevacizumab mechanisms of resistance in mCRC patients,^20^ which was concordant with our data FUT4 in regulating aggressiveness of SW620 and SW480 cells *in vitro* and *in vivo*. Recently, our data also showed FUT4 was crucial regulators of cancer response to chemotherapy in breast cancer and hepatocellular carcinoma, as well as of invasiveness and tumorigenicity in breast cancer.^27, 29, 30^ Thus, miR-26a/26b-induced FUT4 provided a conserved mechanism for the suppressive role of miR-26a/26b during aggressiveness of CRC.

The expression of miR-26a and miR-26b has been reported in several tumors, including osteosarcoma,^33^ hepatocellular carcinoma^34^ and lung carcinoma^35^ and has been identified as a poor prognostic marker in these tumors. In CRC, Jinushi *et al.*,^36^ identified that plasma miR-26a expression level may be used as a prognostic biomarker in CRC. De Robertis *et al.*,^37^ showed that EphA2/Efna1/Egfr genes, linked to a possible control by miR-26b, could be proposed as novel CRC prognostic biomarkers. In this study, we have assessed the expression and prognostic relevance of miR-26a/26b and FUT4 in tissues from CRC patients. A key finding of our study was that low miR-26a/26b expression was significantly associated with poorer overall survival in CRC. Whereas those patients with FUT4 overexpression showed a substantially shorter overall survival as compared to the patients with low FUT4 group. A recent study also reported patients with tumors harboring FUT4-high expression were associated with worse progression-free survival (PFS), indicating FUT4 as a potential prognostic factor for CRC patients.^20^ Therefore, these observations would indicate a potential FUT4-dependent prognostic value for miR-26a/26b which needs to be further confirmed in forthcoming studies. Moreover, we found that the correlation of miR-26a/26b downregulation and FUT4 overexpression was an unfavorable independent factor associated with overall survival in mCRC, and this would be important in the development and refinement of new therapeutic approaches.

In summary, our study defines a mechanism for the suppressive function of miR-26a and miR-26b that directly target FUT4 expression that, in turn, regulates the CSC growth and metastasis. It is possible that targeting miR-26a/26b/FUT4 axis, may improve the outcomes of therapy for patients with CRC.

## Materials and methods

### Cell culture

Human CRC cell lines SW480 and SW620 were obtained from the American Type Culture Collection (ATCC; Manassas, VA, USA). The two cell lines were cultured in Leibovitz’s L-15 (Gibco, Grand Island, NY,USA) medium supplemented with 10% fetal bovine serum (FBS; Gibco, Grand Island, NY, USA), 100 U/ml penicillin, and 100 *μ*g/ml streptomycin (Life Technologies, Cergy Pontoise, France), maintained at 37 °C without CO_2_.

### Clinical samples

The study and its informed consent have been examined and certified by the Ethics Committee of the First Affiliated Hospital of Dalian Medical University. Before collecting tumor specimen written informed consent was acquired from each enrolled patient. All specimens were handled anonymously according to the ethical and legal regulations.

A total of 58 adults (32 males and 26 females; aged from 42 to 79 years) with CRC were enrolled in the current study, from November 2010 to July 2016. Tumor tissues and adjacent tissues (located<3 cm away from the tumor) were obtained from these individuals who had undergone proctocolectomy with lymph node dissection for CRC, at the First Affiliated Hospital of Dalian Medical University (Dalian, China). None of the patients received any chemotherapy or radiation treatment prior to the surgery. Tumor tissues and adjacent tissues were collected after surgical removal and snap-frozen in liquid nitrogen until further use.

### MicroRNA microarray

MicroRNA expression profiles of SW620 group and SW480 group (*n*=3 per group) were generated using the miRCURYHy3/Hy5 power labelling kit and the miRCURY LNA Array (v.10.0; 757 human miRs) by Exiqon (KangChen, China). The expression values are log2 (Hy3/Hy5) ratios. Unsupervised hierarchical clustering of miRNAs was performed.

### RNA extraction and quantitative real-time PCR

Total RNA was isolated from frozen tissues and CRC cell lines, using the RNeasy Mini Kit (QIAGEN, Valencia, CA, USA), and cDNA was synthesized using QuantiTect Reverse Transcription Kit (QIAGEN, valencia, CA, USA) according to the manufacturer’s specifications. The expression of miRNAs was determined by using mirVanaTM qRT-PCR microRNA Detection Kit (Ambion Inc., Austin, TX, USA). Relative quantities of each miRNA were calculated using the ΔΔCt method after normalization with endogenous reference U6-small nuclear RNA. FUT4 mRNA was quantified with SYBR-Green-quantitative real-time PCR Master Mix kit (Toyobo Co., Osaka, Japan). The expression level of FUT4 was determined by using Biosystems 7300 Real-Time PCR system (ABI, Foster City, CA, USA) and calculated using the ΔΔCt method after normalisation with endogenous reference RNA 18 s. All PCR reactions were performed in triplicate for a technical replicate, including no-template controls, and the mean of the triplicates was used.

### Cell transfection

shRNA against FUT4, scrambled shRNA, miR-26a/miR-20b/ normal control (NC) mimics, and miR-26a/miR-26b/NC inhibitors were chemically synthesized by Shanghai GenePharma Co.,Ltd. (Shanghai, China). SW480 and SW620 cells were transfected with miRNAs (100 nM,) or shRNAs (50 nM) using Lipofectamine 2000 Transfection Reagent (Invitrogen).

### Luciferase assay

A pmirGLO Dual-Luciferase miRNA Target Expression Vector was chosen for 3′UTR Luciferase assays (Promega, Madison, WI, USA). The vector could be used to study the influence of miRNAs on transcript stability and activity by the insertion of miRNA target sites 3′ untranslated region (UTR) of gene. The wild-type FUT4 and mutant FUT4 3′-UTR were specifically synthesized (Promega) and inserted into the vector. HEK 293 T cells of 50% confluence were seeded (5 × 10^4^ cells per well) in a 24-well dish and were transfected using Lipofectamine 2000. The miRNA mimic or NC mimic with pmirGLO-FUT4 3′-UTR wt vector, pmirGLO-FUT4 3′-UTR mut vector or pmirGLO vector were co-transfected per well. Luciferase assays were performed up to 48 h after transfection by using the dual luciferase reporter assay system (Promega) according to the manufacturer’s protocol. Luciferase readings were corrected for background, and Firefly and Renilla luciferase activities were measured and normalized to Renilla to control for transfection efficiency. The mean of relative luciferase activities from the cells transfected with the pmirGLO vector and NC mimic was set at 100. The results were presented as the mean value±SD for three repeat experiments.

### Western blot analysis

Samples of equal amounts were separated on SDS-PAGE and transferred onto polyvinylidene difluoride membrane (Pall Corporation). The membrane was blocked with 5% non fat dry milk in PBS containing 0.1% Tween 20 (PBST) for one hour and then probed with anti-FUT4 monoclonal antibody (Abcam, Cambridge, UK, 1:1000 dilution), or anti-GAPDH rabbit polyclonal antibody (Santa Cruz Biotech, Santa Cruz, CA, 1:1000 dilution). Membrane proteins were detected by HRP-conjugated secondary antibody (Santa Cruz Biotech, Santa Cruz, CA, 1:1000 dilution). GAPDH was used as a control. Immunoreactive bands were visualised using ECL Western blotting kit (Amersham Biosciences, UK) and were normalized to those of GAPDH.

### Cell counting kit-8 assay

The cell proliferation assays were performed using cell counting kit-8 (CCK-8; KeyGEN, Nanjing, China) according to the manufacturer’s instruction. Cells (1 × 10^3^ per well) were seeded in 96-well plates with 100 *μ*l of DMEM medium containing 10% FBS and cultured in a humidified incubator (at 37 °C, without CO_2_) for 24, 48 and 72 h, Then, each well was added 10 *μ*l CCK-8 solutions at 37 °C for 2 h. The absorbance at 450 nm was immediately measured using a microplate reader. Each experiment was performed at least 3 times.

### Focus formation assay

To measure focus formation, cells (1 × 10^3^) were trypsinized to single-cell suspension and seeded in six-well plates in. The cultures were maintained in the L-15 containing 10% FBS, with medium changes every 3 days, until the appearance of foci from transformed cells was evident (10 days after transfection). Then the colonies were stained with 0.2% crystal violet, and foci were counted. Images of the colonies were obtained using a NIKON digital camera.

### Immunofluorescence

Cells grown overnight on glass coverslips were washed once with phosphate-buffered saline (PBS), fixed with 3.7% formaldehyde for 30 min, and permeabilized with PBS containing 0.1% Triton X-100 (Sigma) for 30 min. After a wash with PBS, the coverslips were incubated with primary antibody against Ki67 or FUT4 (Abcam, Cambridge, MA, USA) overnight at 4 °C. The coverslips were again washed with PBS, cells were incubated with secondary antibody. The coverslips were washed with PBS and incubated with 1 *μ*g/ml of 4, 6-diamino-2-phenylindole (DAPI, Sigma-Aldrich, St Louis, MO, USA) for nuclear staining. Pictures were taken with fluorescence microscope (OLYPAS).

### Cell invasion assay

Cell invasion assay was performed using transwell inserts with polycarbonate membranes of 8.0 μm pore size (Corning Inc., NY) with ECMatrix gel (Chemicon) to form a continuous thin layer. In brief, 4 × 10^4^ cells in serum-free medium were seeded onto the upper chamber. Culture medium containing 10% FBS was used as a chemoattractant in the lower chamber. Cells were incubated in a humidified incubator at 37 °C for 24 h. Migrated or invaded cells on the lower surface of the membrane were then fixed with methanol, stained with Wright-Giemsa, photographed (× 400) and counted in 5 random fields. Each experiment was performed thrice.

### *In vivo* tumorigenicity assay

To assess the tumorigenicity, cells were trypsinized and resuspended in phosphate-buffered saline. Approximately 1 × 10^7^ Cells were injected subcutaneously into the flank of 5-week-old female athymic nude mice using a 25-gauge needle (*n*=6 for each group of experiments). Tumor size was monitored weekly by measuring the perpendicular tumor diameters, length (L) and width (W). Mice were killed under anesthesia 4 week after injection. Mice were sacrificed and their tumors were isolated, photographed and weighed. Tumor size was measured using calipers and estimated according to the formula: (length × width^2^)/2.

### Tube formation assay

The 96-well plate were coated with cold BD Matrigel (Corning, New York, NY, USA). After incubation of 1 h at 37 °C, Human umbilical vein endothelial cells (HUVECs, 4 × 10^3^ cells per well) were seeded to Matrigel-coated wells and then incubated at 37 °C without CO_2_. Six hour later, three non-overlapping microscopic images in each well were randomly photographed at magnification (× 400). The observed total tube length and branching points formed by endothelial cells per image field were analyzed by using Image J software (National Institutes of Health, Bethesda, MD). The experiment was performed in triplicate and repeated three times.

### Immunohistochemical analysis

For immunohistochemical (IHC) staining, the xenograft tumor was fixed in 4% paraformaldehyde, dehydrated in a graded series of alcohol, and then embedded in paraffin. 3 *μ*m sections were sliced, dried, deparaffinized, rehydrated and then were immersed in 3% hydrogen peroxide for 10 min to block endogenous peroxidase. After consecutive washing with PBS, the slices were incubated with primary anti FUT4 or Ki67 antibody (1:200, Abcam, Cambridge, UK) at 4 °C overnight. The secondary streptavidin-HRP-conjugated antibody staining (Santa Cruz Biotech, Santa Cruz, CA, USA) was performed at room temperature for 60 min. Finally, the sections were counterstained with hematoxylin and cover-slipped. The Image-ProPlus 4.5 Software (Media Cybernetics, USA) was used to analyze the expression of proteins.

### Statistical analysis

Each experiment was performed at least in triplicate, and the measurements were performed in three independent experiments. Data are expressed as means±standard deviation (SD). Student’s *t*-test was used to compare the means of two groups. *P*<0.05 was considered statistically significant. All analyses were performed using SPSS 17.0 statistical packages (SPSS Inc., Chicago, IL).

## Figures and Tables

**Figure 1:** MiRNAs expression profile and identification of miR-26a and miR-26b in CRC cell lines and CRC tissues. (**a**) Microarray chip analysis of miRNAs expression in SW620 and SW480 cells. Columns represented cell lines and rows showed the relative expression level for individual miRNAs. The red and green colors indicated high of low expression, respectively. (**b**) The levels of miR-26a and miR-26b were significantly decreased in metastatic CRC cell SW620 compared with primary CRC cell SW480 by qRT-PCR analysis. (**c**) miR-26a and miR-26b expression was significantly decreased in 38 pairs of CRC tissues compared with the corresponding adjacent noncancerous tissues by qRT-PCR analysis. The experiment was performed in triplicate and repeated three times, and the central horizontal line represented the mean value (*P<0.05)

**Figure 2:** FUT4 is directly modulated by miR-26a and miR-26b negatively. (**a**) The luciferase assays confirmed that miR-26a and miR-26b binds to the wild-type 3′-UTR sequences of FUT4. The nucleotides sequence of the target site of miRNAs in FUT4 3′-UTR were shown. Mut: contains three-base mutation at miR-26a and miR-26b target region. The wide-type and mutant miRNA target sequences of FUT4 were fused with luciferase reporter and transfected into 293T cells, co-transfected with miRNA mimic and NC mimic. The mean of the results from the cells transfected with the NC mimic was set at 100. Each bar represents the relative luciferase activity. (**b**), The mRNA and protein levels of FUT4 in SW620 cells were significantly decreased when SW620 cells were treated with miR-26a mimic, miR-26b mimic and mimic mixture. (**c**) The mRNA and protein levels of FUT4 in SW480 cells were significantly increased when SW480 cells were treated with miR-26a inhibitor, miR-26b inhibitor and inhibitor mixture. Immunofluorescence staining assay shown that levels of FUT4 in SW620 cells were significantly decreased when SW620 cells were treated with miR-26a mimic, miR-26b mimic and mimic mixture (**d**) and levels of FUT4 in SW480 cells were significantly increased when SW480 cells were treated with miR-26a inhibitor, miR-26b inhibitor and inhibitor mixture (**e**). (**f**) The inverse relationship was observed between the expression of miR-26a/-26b and FUT4. (**g**) The mRNA and protein levels of FUT4 in SW480 cells were significantly decreased compared with SW620 cells. (**h**) Comparison on the tissues and cells by IHC and immunofluorescence staining, the significantly lower FUT4 level was observed in adjacent tissues and SW480 cells. The experiment was performed in triplicate and repeated three times, and the central horizontal line represented the mean value (*P<0.05)

**Figure 3:** Effect of miR-26 mimic, miR-26b mimic and mimic mixture on cell aggressiveness in SW480 and SW620 cells. (**a**) CCK-8 assay (**b**) Immunofluorescence staining assay (**c**) colony assay (**e**) wound-healing assay (**g**) transwell assay revealed transfection of miR-26a mimic, miR-26b mimic and mimic mixture in SW620 cells inhibited cellular progression. (**a**) CCK-8 (**b**) Immunofluorescence staining assay (**d**) colony assay (**f**) wound healing assay (**h**) transwell assay revealed transfection of miR-26a inhibitor, miR-26b inhibitor and inhibitor mixture in SW480 cells increased cellular progression. The experiment was performed in triplicate and repeated three times, and the central horizontal line represented the mean value (*P<0.05)

**Figure 4:** FUT4 reverses the effect of miR-26a and miR-26b-mediated CRC cell aggressiveness. (**a** and **b**) The mRNA and protein levels of FUT4 in SW620 miR-26a/26b mimic cells were significantly increased when transfected with FUT4 compared with transfected with mock. (**c** and **d**), Upregulation of FUT4 in SW620 miR-26a/26b mimic cells promoted cellular proliferation and invasion as revealed by colony assay and transwell invasion assay. (**e** and **f**), The mRNA and protein levels of FUT4 in SW480 miR-26a/26b inhibitor cells were significantly decreased when transfected with FUT4 shRNA compared with transfected with NC shRNA. (**g** and **h**), The effect of miR-26a or miR-26b inhibitor on cellular proliferation and invasion was reversed by down-regulation of FUT4 expression in SW480 cells. Values shown are mean±SD from three independent experiments (*P<0.05)

**Figure 5:** Effect of FUT4 on cell invasiveness and tumorigenesis in CRC cell lines. (**a**) The mRNA and protein levels of FUT4 were significantly decreased in SW620 cells by FUT4 shRNA treatment. The ability of proliferation and invasion was compared in SW620 shFUT4 and SW620 control cells based on CCK-8 assay (**b**) and transwell invasion assay (**c**) (*P<0.05). (**d**) Tube formation assay was performed to compare cell tube formation between SW620 shFUT4 cells and control group (*P<0.05). (**e**) A decrease of mean tumor volume in mice group with SW620 shFUT4 tumors was observed, as compared to the control group (*P<0.05). (**f**) Reduced regulation of FUT4 and Ki67 was also shown by IHC staining in xenograft tumors derived from SW620 shFUT4 cells (400 ×). (**g**) After full-length sequences transfection, FUT4 mRNA and protein levels were increased notably in SW480 cells by qRT-PCR and western blot analysis (*P<0.05). CCK-8 assay (**h**) transwell invasion assay (**i**), tube formation assay (**j**) and *in vivo* tumorigenicity assay (**k**) were performed to compare cell progression between SW480 FUT4 cells and SW480 mock. *L*, FUT4 and Ki67 expression was detected by IHC staining in xenograft tumors derived from SW480 FUT4 cells. The data were mean±S.D. of three separate transfections (*P<0.05)

**Figure 6:** Clinical significance of miR-26a, miR-26b and FUT4 in CRC. (**a** and **b**), Kaplan–Meier analysis for overall survival based on miR-26a/26b expression. The red line depicts survival curve for patients with miR-26a/26b low expression levels, and the black line depicts survival curve for patients with miR-26a/26b high expression levels. (**c**) Kaplan–Meier overall survival curves for two groups defined based on low and high FUT4 expression levels. The red curve represents samples that expressed low levels of FUT4, whereas the black curve corresponds to samples that expressed high FUT4 levels. The survival curves were found to be significantly different with a *P* value (*P<0.001)

**Table 1:** Correlation of clinicopathological characteristics with miR-26a expression

	**Total cases (*****N***)	**Relative miR-26a expression**		***P*** **value**
		**Low**	**High**	
Age, years	58	56.66	53.07	0.317
*Gender*				
Male	32	17 (56.67%)	15 (53.57%)	0.813
Female	26	13 (43.33%)	13 (46.43%)	
				
*Stage*				
I–II	27	10 (33.33%)	17 (60.71%)	0.037*
III–IV	31	20 (66.67%)	11 (39.29%)	
				
*Survival*				
Alive	23	3 (10.00%)	20 (71.43%)	0.000*
Dead	35	27 (90.00%)	8 (28.57%)	

*P<0.05

**Table 2:** Correlation of clinicopathological characteristics with miR-26b expression

	**Total cases (*****N***)	**Relative miR-26b expression**		***P*** **value**
		**Low**	**High**	
Age, years	58	55.54	54.44	0.193
*Gender*				
Male	32	14 (58.33%)	18 (52.94%)	0.684
Female	26	10 (41.67%)	16 (47.06%)	
				
*Stage*				
I–II	27	7 (29.17%)	20 (55.88%)	0.026*
III–IV	31	17 (70.83%)	14 (44.12%)	
				
*Survival*				
Alive	23	3 (12.5%)	20 (58.82%)	0.000*
Dead	35	21 (87.5%)	14 (41.18%)	

*P<0.05

**Table 3:** Correlation of clinicopathological characteristics with FUT4 expression

	**Total cases (*****N***)	**Relative FUT4 expression**		***P*** **value**
		**Low**	**High**	
Age, years	58	55.00	54.80	0.955
*Gender*				
Male	32	16 (57.14%)	16 (53.33%)	0.771
Female	26	12 (42.86%)	14 (46.67%)	
				
*Stage*				
I–II	27	17 (60.71%)	10 (33.33%)	0.037*
III–IV	31	11 (39.29%)	20 (66.67%)	
				
*Survival*				
Alive	23	19 (67.86%)	4 (13.33%)	0.000*
Dead	35	9 (32.14%)	26 (86.67%)	

*P<0.05

## References

[bib1] Chen W, Zheng R, Zeng H, Zhang S, He J. Annual report on status of cancer in China, 2011. Chinese J Cancer Res 2015; 27: 2–12.10.3978/j.issn.1000-9604.2015.01.06PMC432917625717220

[bib2] Gill S, Blackstock AW, Goldberg RM. Colorectal cancer. Mayo Clin Proc 2007; 82: 114–129.1728579310.4065/82.1.114

[bib3] Weitz J, Koch M, Debus J, Hohler T, Galle PR, Buchler MW. Colorectal cancer. Lancet (London, England) 2005; 365: 153–165.10.1016/S0140-6736(05)17706-X15639298

[bib4] Bartel DP. MicroRNAs: genomics, biogenesis, mechanism, and function. Cell 2004; 116: 281–297.1474443810.1016/s0092-8674(04)00045-5

[bib5] Mitchell PS, Parkin RK, Kroh EM, Fritz BR, Wyman SK, Pogosova-Agadjanyan EL et al. Circulating microRNAs as stable blood-based markers for cancer detection. Proc Natl Acad Sci USA 2008; 105: 10513–10518.1866321910.1073/pnas.0804549105PMC2492472

[bib6] Chen X, Ba Y, Ma L, Cai X, Yin Y, Wang K et al. Characterization of microRNAs in serum: a novel class of biomarkers for diagnosis of cancer and other diseases. Cell Res 2008; 18: 997–1006.1876617010.1038/cr.2008.282

[bib7] Friedman RC, Farh KK, Burge CB, Bartel DP. Most mammalian mRNAs are conserved targets of microRNAs. Genome Res 2009; 19: 92–105.1895543410.1101/gr.082701.108PMC2612969

[bib8] Gattolliat CH, Uguen A, Pesson M, Trillet K, Simon B, Doucet L et al. MicroRNA and targeted mRNA expression profiling analysis in human colorectal adenomas and adenocarcinomas. Eur J Cancer 2015; 51: 409–420.2558694410.1016/j.ejca.2014.12.007

[bib9] Bandres E, Cubedo E, Agirre X, Malumbres R, Zarate R, Ramirez N et al. Identification by Real-time PCR of 13 mature microRNAs differentially expressed in colorectal cancer and non-tumoral tissues. Mol Cancer 2006; 5: 29.1685422810.1186/1476-4598-5-29PMC1550420

[bib10] Meng WJ, Yang L, Ma Q, Zhang H, Adell G, Arbman G et al. MicroRNA Expression Profile Reveals miR-17-92 and miR-143-145 Cluster in Synchronous Colorectal Cancer. Medicine 2015; 94: e1297.2626636610.1097/MD.0000000000001297PMC4616700

[bib11] Okugawa Y, Toiyama Y, Goel A. An update on microRNAs as colorectal cancer biomarkers: where are we and what's next? Expert Rev Mol Diagn 2014; 14: 999–1021.2516335510.1586/14737159.2014.946907PMC4374444

[bib12] Yang IP, Tsai HL, Huang CW, Huang MY, Hou MF, Juo SH et al. The functional significance of microRNA-29c in patients with colorectal cancer: a potential circulating biomarker for predicting early relapse. PLoS ONE 2013; 8: e66842.2384053810.1371/journal.pone.0066842PMC3696003

[bib13] Bertozzi CR, Kiessling LL. Chemical glycobiology. Science 2001; 291: 2357–2364.1126931610.1126/science.1059820

[bib14] Khoury GA, Baliban RC, Floudas CA. Proteome-wide post-translational modification statistics: frequency analysis and curation of the swiss-prot database. Sci Rep 2011; 1: srep00090.2203459110.1038/srep00090PMC3201773

[bib15] Sethi MK, Hancock WS, Fanayan S. Identifying N-glycan biomarkers in colorectal cancer by mass spectrometry. Acc Chem Res 2016; 49: 2099–2106.2765347110.1021/acs.accounts.6b00193

[bib16] Holst S, Deuss AJ, van Pelt GW, van Vliet SJ, Garcia-Vallejo JJ, Koeleman CA et al. N-glycosylation profiling of colorectal cancer cell lines reveals association of fucosylation with differentiation and caudal type homebox 1 (CDX1)/Villin mRNA expression. Mol Cell Proteomics 2016; 15: 124–140.2653779910.1074/mcp.M115.051235PMC4762531

[bib17] Osuga T, Takimoto R, Ono M, Hirakawa M, Yoshida M, Okagawa Y et al. Relationship between increased fucosylation and metastatic potential in colorectal cancer. J Nstl Cancer Inst 2016; 108: djw210.10.1093/jnci/djw21027628655

[bib18] Aziz F, Gao W, Yan Q. Fucosyltransferase-4 and oligosaccharide Lewis Y antigen as potentially correlative biomarkers of Helicobacter pylori CagA associated gastric cancer. Pathol Oncol Res 2017; 23: 173–179.2775783810.1007/s12253-016-0122-1

[bib19] Yang X, Liu S, Yan Q. Role of fucosyltransferase IV in epithelial-mesenchymal transition in breast cancer cells. Cell Death Dis 2013; 4: e735.2388762610.1038/cddis.2013.241PMC3730415

[bib20] Giordano G, Febbraro A, Tomaselli E, Sarnicola ML, Parcesepe P, Parente D et al. Cancer-related CD15/FUT4 overexpression decreases benefit to agents targeting EGFR or VEGF acting as a novel RAF-MEK-ERK kinase downstream regulator in metastatic colorectal cancer. J Exp Clin Cancer Res 2015; 34: 108.2642791410.1186/s13046-015-0225-7PMC4590269

[bib21] Cheng L, Luo S, Jin C, Ma H, Zhou H, Jia L. FUT family mediates the multidrug resistance of human hepatocellular carcinoma via the PI3K/Akt signaling pathway. Cell Death Dis 2013; 4: e923.2423209910.1038/cddis.2013.450PMC3847326

[bib22] Slattery ML, Herrick JS, Pellatt DF, Mullany LE, Stevens JR, Wolff E et al. Site-specific associations between miRNA expression and survival in colorectal cancer cases. Oncotarget 2016; 7: 60193–60205.2751762310.18632/oncotarget.11173PMC5312378

[bib23] Konishi H, Fujiya M, Ueno N, Moriichi K, Sasajima J, Ikuta K et al. microRNA-26a and -584 inhibit the colorectal cancer progression through inhibition of the binding of hnRNP A1-CDK6 mRNA. Biochem Biophys Res Commun 2015; 467: 847–852.2649429910.1016/j.bbrc.2015.10.055

[bib24] Wang M, Wang J, Kong X, Chen H, Wang Y, Qin M et al. MiR-198 represses tumor growth and metastasis in colorectal cancer by targeting fucosyl transferase 8. Sci Rep 2014; 4: 6145.2517445010.1038/srep06145PMC5385833

[bib25] Bernardi C, Soffientini U, Piacente F, Tonetti MG. Effects of microRNAs on fucosyltransferase 8 (FUT8) expression in hepatocarcinoma cells. PLoS ONE 2013; 8: e76540.2413078010.1371/journal.pone.0076540PMC3793929

[bib26] Wu CS, Yen CJ, Chou RH, Chen JN, Huang WC, Wu CY et al. Downregulation of microRNA-15b by hepatitis B virus X enhances hepatocellular carcinoma proliferation via fucosyltransferase 2-induced Globo H expression. Int J Cancer 2014; 134: 1638–1647.2412237510.1002/ijc.28501

[bib27] Cheng L, Gao S, Song X, Dong W, Zhou H, Zhao L et al. Comprehensive N-glycan profiles of hepatocellular carcinoma reveal association of fucosylation with tumor progression and regulation of FUT8 by microRNAs. Oncotarget 2016; 7: 61199–61214.2753346410.18632/oncotarget.11284PMC5308645

[bib28] Li N, Liu Y, Miao Y, Zhao L, Zhou H, Jia L. MicroRNA-106b targets FUT6 to promote cell migration, invasion, and proliferation in human breast cancer. IUBMB Life 2016; 68: 764–775.2751916810.1002/iub.1541

[bib29] Feng X, Zhao L, Gao S, Song X, Dong W, Zhao Y et al. Increased fucosylation has a pivotal role in multidrug resistance of breast cancer cells through miR-224-3p targeting FUT4. Gene 2016; 578: 232–241.2670161510.1016/j.gene.2015.12.028

[bib30] Zhao L, Feng X, Song X, Zhou H, Zhao Y, Cheng L et al. miR-493-5p attenuates the invasiveness and tumorigenicity in human breast cancer by targeting FUT4. Oncol Rep 2016; 36: 1007–1015.2737504110.3892/or.2016.4882

[bib31] Chen B, Liu Y, Jin X, Lu W, Liu J, Xia Z et al. MicroRNA-26a regulates glucose metabolism by direct targeting PDHX in colorectal cancer cells. BMC Cancer 2014; 14: 443.2493522010.1186/1471-2407-14-443PMC4071217

[bib32] Zhang C, Tong J, Huang G. Nicotinamide phosphoribosyl transferase (Nampt) is a target of microRNA-26b in colorectal cancer cells. PLoS ONE 2013; 8: e69963.2392287410.1371/journal.pone.0069963PMC3726743

[bib33] Song QC, Shi ZB, Zhang YT, Ji L, Wang KZ, Duan DP et al. Downregulation of microRNA-26a is associated with metastatic potential and the poor prognosis of osteosarcoma patients. Oncol Rep 2014; 31: 1263–1270.2445259710.3892/or.2014.2989

[bib34] Yang X, Liang L, Zhang XF, Jia HL, Qin Y, Zhu XC et al. MicroRNA-26a suppresses tumor growth and metastasis of human hepatocellular carcinoma by targeting interleukin-6-Stat3 pathway. Hepatology (Baltimore, Md) 2013; 58: 158–170.10.1002/hep.2630523389848

[bib35] Gao W, Shen H, Liu L, Xu J, Xu J, Shu Y. MiR-21 overexpression in human primary squamous cell lung carcinoma is associated with poor patient prognosis. J Cancer Res Clin Oncol 2011; 137: 557–566.2050894510.1007/s00432-010-0918-4PMC11828261

[bib36] Jinushi T, Shibayama Y, Kinoshita I, Oizumi S, Jinushi M, Aota T et al. Low expression levels of microRNA-124-5p correlated with poor prognosis in colorectal cancer via targeting of SMC4. Cancer Med 2014; 3: 1544–1552.2508186910.1002/cam4.309PMC4298381

[bib37] De Robertis M, Loiacono L, Fusilli C, Poeta ML, Mazza T, Sanchez M et al. Dysregulation of EGFR pathway in EphA2 cell subpopulation significantly associates with poor prognosis in colorectal cancer. Clin Cancer Res 2017; 23: 159–170.2740124810.1158/1078-0432.CCR-16-0709PMC5822042

